The article "A Retrospective Study: Quick Scoring of Symptoms to Estimate the Risk of Cardiac Arrest in the Emergency Department" was published in 2022. Journal: Emerg Med Int.

# A Retrospective Study: Quick Scoring of Symptoms to Estimate the Risk of Cardiac Arrest in the Emergency Department

**DOI:** 10.1155/2022/6889237

**Published:** 2022-11-18

**Authors:** Yaoke Xu, Hua Zhang, Zongxuan Zhao, Kaifeng Wen, Ci Tian, Qiangrong Zhai, Yi Bai, Shu Li, Hongxia Ge, Xiaodan Li, Qidi Zhou, Qingbian Ma

**Affiliations:** ^1^Emergency Department, The Peking University Third Hospital, No. 49 North 9 Garden Road, Haidian District, Beijing 100191, China; ^2^Research Center of Clinical Epidemiology, Peking University Third Hospital, Beijing 19, China; ^3^Emergency Department, Peking University Shenzhen Hospital, 1120 Lianhua 20 Road, Futian District, Shenzhen City 518306, Guangdong, China

## Abstract

**Purpose:**

At present, not enough is known about the symptoms before cardiac arrest. The purpose of this study is to describe the precursor symptoms of cardiac arrest, focusing on the relationship between symptoms and cardiac arrest, and to establish a quick scoring model of symptoms for predicting cardiac arrest. *Patients and Methods*. A retrospective case-control study was carried out on cardiac arrest patients who visited the emergency department of Peking University Third Hospital from January 2018 to June 2019. Symptoms that occurred or were obviously aggravated within the 14 days before CA were defined as warning symptoms.

**Results:**

More than half the cardiac arrest patients experienced warning symptoms within 14 days before cardiac arrest. Dyspnea (*p* < 0.001) was found to be associated with cardiac arrest; syncope and cold sweat are other symptoms that may have particular clinical significance. Gender (*p* < 0.001), age (*p* < 0.001), history of heart failure (*p*=0.006), chronic kidney disease (*p*=0.011), and hyperlipidemia (*p*=0.004) were other factors contributing to our model.

**Conclusions:**

Warning symptoms during the 14 days prior to cardiac arrest are common for CA patients. The Quick Scoring Model for Cardiac Arrest (QSM-CA) was developed to help emergency physicians and emergency medical services (EMS) personnel quickly identify patients with a high risk of cardiac arrest.

## 1. Introduction

Cardiac arrest (CA) refers to the sudden termination of cardiac ejection that result in interruption of systemic blood circulation, respiratory arrest, and loss of consciousness [1]. As a potentially fatal cardiovascular event with poor prognosis, especially when it occurs outside of a hospital, CA has become a public health threat around the world. It is generally accepted that 4–6 minutes after the occurrence is the ideal time for treatment. However, there are several early warning symptoms of cardiac arrest, including chest pain, dyspnea, syncope, cold sweat, backache, abdominal pain, and palpitation [2, 3], and the presence of these prodromal symptoms could persuade people to contact their doctors early enough to prevent cardiac arrest [4] if the public were aware of them. Yet no effective early warning model has been broadly employed, though it is of great significance to identify the high-risk population and provide timely warning of imminent cardiac arrest. Establishing a warning model based on prodromal symptoms would earn time for prevention and intervention of out-of-hospital cardiac arrest [5] by emergency medical services (EMS), and could ultimately promote public awareness. This study explored the correlations between CA and warning symptoms and therefore developed a symptoms-based quick scoring model for CA using one and a half years of emergency room data.

The article "A Retrospective Study: Quick Scoring of Symptoms to Estimate the Risk of Cardiac Arrest in the Emergency Department" was published in 2022. Journal: Emerg Med Int.

## 2. Materials and Methods

### 2.1. Patients and Study Design

This single-center retrospective case-control study was conducted at Peking University Third Hospital, which has about 240,000 emergency visits per year. From January 2018 to June 2019, we extracted data for 309 consecutive cardiac arrest (CA) patients. The incidence of cardiac arrest was defined as the cessation of mechanical cardiac activity as confirmed by the absence of signs of circulation.

A total of 150 patients over 18 years old were enrolled in the case group after excluding patients with a history of trauma, drug overdose, drowning, pregnancies, end-stage malignancies, and patients with severe instances of missing data. Patients who were pronounced clinically dead before admission were also excluded because of the low proportion of sudden CAs, as confirmed by autopsy. All enrolled patients had detailed records of rescue and short-term outcomes after CA. Of the case group, 98 were out-of-hospital cardiac arrest (OHCA) and 52 were in-hospital CA (IHCA). A control group of noncardiac arrest patients who visited the emergency department on the same date were randomly enrolled in a 1 : 3 ratio, totaling 450 cases in the control group. The exclusion criteria for the case group were also used for the control group. Patients in a perioperative period were also excluded from the control group.

### 2.2. Data Collection

Data were collected from the electronic health records of Peking University Third Hospital by three authorized researchers on standard forms and double keyed into an Epidata 3.1 database (Odense, Denmark). The case report form was designed based on the Utstein-style uniform guidelines for out-of-hospital CA, which includes the patient variables, arrest variables, prodromal symptoms and outcomes [6] shown in Table 1.

The article "A Retrospective Study: Quick Scoring of Symptoms to Estimate the Risk of Cardiac Arrest in the Emergency Department" was published in 2022. Journal: Emerg Med Int.

Identification of the conditions underlying CA is one of the interests of this study, which, according to previous research, includes age, cardiovascular diseases, respiratory diseases, and diabetes. Close attention was paid to patients' history of smoking and drinking. Symptoms that occurred or were obviously aggravated within 14 days before CA were defined as prodromal symptoms. All symptoms were recorded, with particular attention to dyspnea, chest pain, abdominal pain, backache, syncope, cold sweat, and palpitation [7]. Data on the duration and character of the symptoms were also collected [8].

The primary outcome of this study was the incidence of cardiac arrest. Gender, age, underlying diseases, and early warning symptoms and were included in the model for clinical use.

### 2.3. Statistical Analysis

R4.0.3 statistical software was used for statistical analysis. The LRM function was used to perform binary logistic regression analysis. When the independent variable was the classification variable, the minimum value group was taken as the reference group. When the independent variable is a continuous variable, the continuous variable is directly included in the binary logistic regression model. The enter regression was used to screen variables, and the nomogram and calibration curve were made. The pROC package was used to draw the ROC curve. A *p* value < 0.05 was considered statistically significant. Different combinations were set up according to statistical stability and the researchers' clinical experience. Five-fold cross-validation was used for model evaluation.

## 3. Results

### 3.1. Epidemiological and Clinical Characteristics of Cardiac Arrest Patients

The patient enrollment flow is shown in Figure 1. Of the 150-patient case group, 98 were OHCA and 52 were in-hospital cardiac arrest (IHCA). All 35 patients in the case group survived to discharge. Though only 22 (22.4%) of the 98 OHCA patients had bystander CPR, OHCA patients had a 28.6% (*n* = 28) return of spontaneous circulation (ROSC), and a discharge survival rate of 23.5% (*n* = 23). A comparison of demographic and clinical characteristics between the cardiac arrest group and control group is shown in Table 2. Patients who suffered from cardiac arrest had more incidence of underlying disease than the control group.

We also presented several important clinical predictors and factors with statistical significance (Table 2), which indicates that more than half of the CA patients suffered from prodromal symptoms. The seven listed symptoms are considered potential risk factors based on previous research: dyspnea, chest pain, abdominal pain, backache, syncope, cold sweat, and palpitation [4]. This study found four of them to show no significance, but dyspnea, syncope, and cold sweat were found to be related to cardiac arrest.

The article "A Retrospective Study: Quick Scoring of Symptoms to Estimate the Risk of Cardiac Arrest in the Emergency Department" was published in 2022. Journal: Emerg Med Int.

### 3.2. Risk Factors and the Quick Scoring Model for Cardiac Arrest

Factors with statistical significance were included as independent variables to explore risk factors. Logistic regression analysis was used to select which independent variables were most suitable for the model. Our results concurred with previous research [6] in finding that cardiac arrest is associated with gender, age, and three of the previously tested diseases. We also found dyspnea is another independent risk factor. Although stroke showed a significant correlation, it was not included in our model considering the small samples. The model thus includes six independent risk factors: gender, age, heart failure history, chronic kidney disease, hyperlipidemia, and dyspnea (Table 3). The characteristics of cardiac arrest patients in the emergency department can be well described by this model, which became our new scoring model, the Quick Scoring Model for Cardiac Arrest (QSM-CA), for emergency room physicians to identify high cardiac arrest risk patients early.

With logistic analysis, we were able to assign values to each of the variables (shown in Table 3) and total them as a predictive risk score. The prediction model was constructed by nomograph (Figure 2). The AUC (C Index) of the area under the ROC curve was calculated to be 0.834. One of the standard methods for evaluating a model is through five-fold cross-validation. The results of all the folds are combined and reported. Sensitivity and specificity were 39% and 95%, respectively, and the AUC was 0.829.

### 3.3. Symptoms

Table 4 indicates the frequency of prodromal symptoms according to the time from its onset to CA. Among 90 patients with prodromes, 48 (32%) patients went through dyspnea. The average elapsed time from the onset of prodromes to cardiac arrest is 39.13 hours while over half the prodromal symptoms (59.0%) occurred within 24 hours of CA.

## 4. Discussion

The incidence of OHCA in adults is 100.1/100,000 per year in Beijing, of which only 19.7% received cardiopulmonary resuscitation provided by emergency centers, and only 1.3% survived [9]. Because this study did not include pre-hospital deaths, our survival rate of 23.5% is higher than in some other studies. Referring to previous studies on early warning symptoms before cardiac arrest, we selected dyspnea, chest pain, abdominal pain, back pain, syncope, cold sweat, and palpitation [7, 10]. Nearly, 61% of the 150 patients in the current study had early warning or prodrome symptoms within 2 weeks before CA, which matches with Binz and Andrea [10] (56%). In our study, more than 50% of the symptoms occurred within 24 hours of CA, as shown in (Table 4). These findings highlight the potential for developing a new model base on consideration of warning symptoms.

The article "A Retrospective Study: Quick Scoring of Symptoms to Estimate the Risk of Cardiac Arrest in the Emergency Department" was published in 2022. Journal: Emerg Med Int.

The incidence rate of Korean prodrome is almost the same as domestic statistics [7]. Compared with previous studies, the incidence of chest pain before cardiac arrest was 3.33%, lower than the Japanese study (20.7%) and another study (48.8%). While the incidence of dyspnea was 32%, higher than in the Japanese study and similar to another studies. Syncope (3.3%) was slightly less common, and cold sweat (8.7%) was more common.

As for the selection of the control group, it is difficult to select the perfect control group because the probability of symptoms before cardiac arrest is very low in healthy people and requires a large sample size. Therefore, we selected the population of outpatient emergency treatment as the control group, whose population is suitable for the medical applications (people who have some health problems).

The model has great predictive value for cardiac arrest and the AUC was 0.834, which includes age, gender, underlying disease, and symptoms [9]. The underlying diseases found to be associated with cardiac arrest were consistent with previous studies, including acute myocardial infarction, cerebrovascular disease, hypertension, heart failure, diabetes, chronic kidney disease, hyperlipidemia, and asthma. Only heart failure, chronic kidney disease, and hyperlipidemia contributed to the model. Diabetes and hypertension in the CA group (35.4% and 57.85%) and control group (18.24% and 33.62%) have a high prevalence rate in both CA, and are often accompanied by other symptoms, so it has not been included in the model. In order to improve the specificity of the model and recognize deteriorating patients, we finally chose not to include these basic diseases. According to previous research, a healthy lifestyle might reduce the risk of cardiac arrest [11]. Our study shows that both smoking history and alcohol history are risk factors for CA, but neither contributed to the model because a lack of ongoing records on these factors might cause systematic error and selection bias. The conclusions of this research still need further confirmation and amendment by relevant studies.

We found that the incidence rate of chest pain and palpitation is very low. The possible reasons are as follows: first, because not all selected patients with CA are cardiogenic, of which cardiogenic accounts for 41.3% and noncardiogenic accounts for 58.6%; second, palpitation and chest pain, as subjective symptoms, are difficult to obtain after cardiac arrest. Dyspnea, as a symptom that can be observed and recorded by bystanders, appears more frequently in the main complaint. In the process of incorporating symptoms into the model, due to changes in consciousness and seizures often accompanied by dyspnea, they were not included in the model at last.

The article "A Retrospective Study: Quick Scoring of Symptoms to Estimate the Risk of Cardiac Arrest in the Emergency Department" was published in 2022. Journal: Emerg Med Int.

The study has several strengths. The model could improve the stratification of patients, enabling more immediate action for those known to be at higher risk to prevent further deterioration because most patients have antecedents before the attack and early intervention is associated with decreased unexpected cardiac arrests and unexpected deaths according to Chen's research [12].

The combination of multiple laboratory tests and vital sign observations are used to develop predictive models such as National Early Warning Score (NEWS) [13]. In addition, the Modified Early Warning Score (MEWS) [14] and the electronic Cardiac Arrest Risk Triage (eCART) score [15] have been investigated in a number of previous studies dealing with in-hospital patients [16]. These scoring methods, however, use CA variables that rely on accurate laboratory examination results and continuous monitoring of vital signs [17], which are difficult to obtain for OHCA. The innovation of our Quick Score Model for Cardiac Arrest (QSM-CA) is that it is based on simple warning symptoms that can be quickly acquired in short conversations with patients or their families in an emergency department or EMS. This model is thus a useful tool to identify those at high CA risk and is applicable to the emergency environment.

It is the first study in which warning symptoms are included as predictive factors. Strong correlations were found between several symptoms such as dyspnea, syncope, cold sweat, and cardiac arrest. Although we had an insufficient number of samples of syncope and cold sweat in this experiment, the models in which they were included showed remarkable predictability. Despite the inadequate sample, the results still have some clinical value for subsequent research. Vettor's research also suggested exercise-induced syncope as an important and alarming symptom of arrhythmic cardiac arrest [18]. Syncope and cold sweat were incorporated into two other models, however, both of them were unstable. Surprisingly, neither chest pain nor the different nature of chest pain showed significance in our study. With only 5 chest pains (3.33%) reported before CA in our study, which is markedly lower than previous studies (22%–48%) [3, 19], it is far too risky to draw conclusive from one set of results.

This study has a few other limitations as well. It was a single-center retrospective study with limited data sources, all the data coming from the clinical records of emergency department patients. Due to the urgent circumstances characteristic of that environment, emergency medical personnel may not be able to identify all symptoms in the process of data collection. As the prediction factors included in the model are limited, any incomplete clinical information could cause migration error. Records of symptoms were also somewhat general; symptoms of different severity and nature can represent totally different clinical significance. For example, severe persistent primordial pain shows a higher predictive value for CA than does chest pain caused by cough. As no consensus is available on the definitions of some of the other warning symptoms, they can be challenged, which could have led to overestimation of their incidence in this study.

The article "A Retrospective Study: Quick Scoring of Symptoms to Estimate the Risk of Cardiac Arrest in the Emergency Department" was published in 2022. Journal: Emerg Med Int.

Electronic in-hospital patient safety net systems like between the Flags have improved the early recognition of deteriorating patients [13] and the reduction in CA and CA-related mortality [20]. One of the challenges with any out-of-hospital health monitoring system is timely emergency calls from patients, families, or by-standers. Simple health warning systems embedded in personal terminals are necessary. Taking the occurrence of symptoms into account can help people decide when to seek help, such as whether to go to the emergency room or call emergency services. Our model initially shows the feasibility of establishing an out-of-hospital early warning system. It also helps EMS identify patients at high risk of CA and can be applied to the triage of patients in an emergency department.

In our next step in this experimental research, we plan to use EMS testing with current clinical data to validate and modify the model, which will be conducive to further development and improvement of the future application.

## 5. Conclusions

More than half of the patients in this study experienced warning symptoms within 24 hours before cardiac arrest. Dyspnea, syncope, and cold sweat may have specific significance in patients presenting to an emergency department. The Quick Score Model for Cardiac Arrest (QSM-CA) is set up by a combination of six independent risk factors: gender, age, heart failure history, chronic kidney disease, hyperlipidemia, and dyspnea, which helps with the timely identification of patients with high risk of cardiac arrest.

## Figures and Tables

**Figure 1:** The patients' enrollment.

**Figure 2:** (a) Nomograph of the QSM-CA model, we assign values to each of the variables (Table 3) and total them as a predictive risk score. (b) ROC of the model, the AUC (C index) of the area under the ROC curve was 0.834.

The article "A Retrospective Study: Quick Scoring of Symptoms to Estimate the Risk of Cardiac Arrest in the Emergency Department" was published in 2022. Journal: Emerg Med Int.

**Table 1:** Variables collected from the electronic health records of Peking University Third Hospital.

*Patient variables*	Age
	Gender
	Hospitalization information such as time of first medical contact and visiting pattern
	Underlying diseases

*Arrest variables*	Vital signs before CA, including temperature, heart rate, blood pressure, and blood oxygen saturation
	Laboratory tests such as routine blood test, coagulation function, and inflammatory factors
	Exact time and location of the attack
	Initial ECG rhythms (shockable rhythm and nonshockable rhythm)
	Witness or bystander CPR
	Rescue measures, including CPR, defibrillation, auxiliary ventilation, and resuscitation drugs

*Outcome variables*	Admission survival, ROSC, and survival to discharge
	Neurological outcome at discharge
	Presumed etiology of CA or preliminary diagnosis of non-CA patients

*Prodromal symptoms*	Dyspnea, chest pain, abdominal pain, backache, syncope, cold sweat, and palpitation

**Table 2:** Epidemiological and clinical characteristics of the study patients.

	N-CA (*n* = 450)	CA (*n* = 150)	*χ* ^2^/*z*	*p*
*Gender*			34.593	<0.001
Female	208 (46.33%)	111 (74%)		
Male	241 (53.67%)	39 (26%)		

Age	51 (32, 69)	66 (51, 78)	−5.946	<0.001
Cerebrovascular diseases	137 (33.58%)	73 (54.89%)	19.177	<0.001
Coronary heart disease	45 (13.85%)	44 (38.6%)	31.986	<0.001
Heart failure	8 (2.62%)	18 (17.48%)	28.469	<0.001
Hypertension	119 (33.62%)	70 (57.85%)	22.108	<0.001
*Respiratory disease*	6 (1.99%)	10 (9.9%)	10.445	0.001

Asthma	6 (1.98%)	7 (6.86%)	4.389	<0.001
Chronic renal diseases	11 (3.58%)	18 (17.14%)	21.985	<0.001
Hyperlipidemia	18 (5.77%)	20 (19.05%)	16.724	<0.001
Diabetes mellitus	60 (18.24%)	40 (35.4%)	14.15	<0.001
Other disease	38 (12.62%)	32 (32%)	19.556	<0.001
Smoking history	1 (0.33%)	19 (19%)	51.504	<0.001
Drinking history	1 (0.33%)	14 (13.86%)	34.982	<0.001

*Symptoms* ^*∗*^	280 (65.57%)	90 (60.81%)	1.087	0.297
Chest pain	39 (8.67%)	5 (3.33%)	4.709	0.03
Dyspnea	36 (8%)	48 (32%)	53.821	<0.001
Palpitation	18 (4%)	4 (2.67%)	0.566	0.452
Abdominal pain	69 (15.3%)	4 (2.67%)	16.891	<0.001
Backache	15 (3.33%)	4 (2.67%)	0.018	0.893
Syncope	3 (0.7%)	5 (3.3%)	6.081	0.026
Cold sweat	2 (0.4%)	13 (8.7%)	31.202	<0.001
Chest tightness	19 (6.23%)	12 (11.43%)	3.021	0.082
Nausea	23 (7.49%)	10 (9.62%)	0.474	0.491
Vomit	29 (9.42%)	15 (14.02%)	1.775	0.183
Altered level of consciousness	2 (0.66%)	6 (6%)	8.408	0.004
Dizziness	43 (13.78%)	10 (9.9%)	1.027	0.311
Seizure	0 (0%)	5 (5%)	11.45	0.001
Other symptoms	0 (0%)	4 (3.88%)	8.177	0.004

^*∗*^a patient may have more than one symptom at the same time.

**Table 3:** Quick scoring model for CA.

		B	SE	*z*	*p*	Or [95% CI]
CA	*Age*	0.026	0.007	3.724	<0.001	1 [1, 1]
	＜35	Ref				
	35∼64	1.056	0.342	3.086	0.002	2.88 [1.47, 5.63]
	≥65 y	1.509	0.344	4.390	0.000	4.52 [2.31, 8.87]
	Male	1.244	0.233	5.336	0.000	3.47 [2.2, 5.48]
	Heart failure	1.368	0.490	2.790	0.005	3.93 [1.5, 10.27]
	Chronic kidney disease	1.01	0.443	2.280	0.023	2.75 [1.15, 6.55]
	Hyperlipidemia	0.761	0.391	1.947	0.052	2.14 [1, 4.6]
	Dyspnea	1.149	0.275	4.177	0.000	3.15 [1.84, 5.41]
	Constant	−3.292	0.347	−9.484	0.000	

Table 3: Six independent risk factors are included in the model: gender, age, heart failure history, chronic kidney disease, hyperlipidemia, and dyspnea. As for age, patients are divided into three groups according to their age, and the group in column 1 (age < 35) is used as the reference index in the model.

The article "A Retrospective Study: Quick Scoring of Symptoms to Estimate the Risk of Cardiac Arrest in the Emergency Department" was published in 2022. Journal: Emerg Med Int.

**Table 4:** The interval from prodromal symptoms to CA.

Prodromal symptoms	Time from symptoms to cardiac arrest			*N* of CA ^*∗*^	Discharge survival
	14 days to 24 hours	2 hours to 24 hours	≤2 hours		
Dyspnea	14	14	6	48 (32%)	9 (18.8%)
Chest pain	2	2	0	5 (3.33%)	0 (0%)
Abdominal pain	0	0	0	4 (2.67%)	0 (0%)
Backache	0	0	2	4 (2.67%)	2 (50%)
Syncope	3	1	0	5 (3.33%)	3 (60%)
Cold sweat	4	7	2	13 (8.67%)	0 (0%)
Palpitation	2	0	2	4 (2.67%)	1 (25%)
Others ^*∗*^				32 (21.33%)	13 (40.6%)
Nonsymptoms ^*∗*^				34 (22.67%)	6 (17.6%)

## Data Availability

The characteristics of patients data used to support the findings of this study have not been made available because the data contains personal information on human subjects.
